The article "High-Throughput Screening and Molecular Dynamics Simulation of Natural Products for the Identification of Anticancer Agents against MCM7 Protein" was retracted in 2023. Reasons: signs of a paper mill; suspected computer-generated content; unreliable results or conclusions; concerns about the data.

# High-Throughput Screening and Molecular Dynamics Simulation of Natural Products for the Identification of Anticancer Agents against MCM7 Protein

**DOI:** 10.1155/2022/8308192

**Published:** 2022-09-15

**Authors:** Xin Zhang, Hui Chen, Hui Lin, Ronglan Wen, Fan Yang

**Affiliations:** Breast Surgery Department, Affiliated Fuzhou First Hospital of Fujian Medical University, Fuzhou 350009, China

## Abstract

Minichromosome maintenance complex component 7 (MCM7) belongs to the minichromosome maintenance family that is necessary for the initiation of eukaryotic DNA replication. Overexpression of the MCM7 protein is linked to cellular proliferation and is accountable for critical malignancy in many cancers. Mechanistically, the suppression of MCM7 greatly lowers the cellular proliferation associated with cancer. Advances in immunotherapy have revolutionized treatments for many types of cancer. To date, no effective small molecular candidate has been found that can stop the advancement of cancer produced by the MCM7 protein. Here, we present the findings of methods that used a combination of structure-assisted drug design, high-throughput virtual screening, and simulations studies to swiftly generate lead compounds against MCM7 protein. In the current study, we designed efficient compounds that may combat all emerging cancer targeting the common MCM7 protein. For this objective, a molecular docking and molecular dynamics (MD) simulation-based virtual screening of 29,000 NPASS library was carried out. As a consequence of using specific pharmacological, physiological, and ADMET criteria, four new prevailing compounds, NPA000018, NPA000111, NPA00305, and NPA014826, were successfully selected. The MD simulations were also used for a time period of 50 ns to evaluate for stability and dynamics behavior of the compounds. Eventually, compounds **NPA000111** and **NPA014826** were found to be highly potent against MCM7 protein. According to our results, the selected compounds may be effective in treating certain cancer subtypes, for which additional follow-up experimental validation is recommended.

## 1. Introduction

Cancer is still a leading cause of death across the globe, despite significant attempts to treat it. Cancer is thought to be caused by the distortion of a normal cell-mediated by DNA mutations and malfunction [1]. These abnormal cells with defective functions bypass the arriving regulatory information needed for proper cellular proliferation and hence multiply, progress, and invade irregularly [1]. At some point in the progression of this aberrant expansion, the tumor microenvironment (TME) is formed, which is a favorable milieu for cancer cells to invade surrounding cells and tissues [2, 3]. It is possible to target various components of the cancer cell's molecular machinery for promising intervention [4–6].

The article "High-Throughput Screening and Molecular Dynamics Simulation of Natural Products for the Identification of Anticancer Agents against MCM7 Protein" was retracted in 2023. Reasons: signs of a paper mill; suspected computer-generated content; unreliable results or conclusions; concerns about the data.

Predicting future cancer cases and fatalities, the Global Cancer Observatory (GLOBOCAN) forecasts 19.3 million new cancer diagnoses in 2020 and about 10.0 million cancer-related deaths globally [7]. The most lethal malignancies were lung cancer, which affects 1.8 million individuals worldwide and accounts for 18% of all cancer fatalities, whereas colon, liver, stomach, and female breast cancer claimed around 9.4%, 8.3%, 7.7%, and 6.9% of lives globally, respectively [7]. Globally, the death rate continues to rise as a result of aging and population growth [8, 9]. Currently, Asia contributes to 48% of the total number of new cancer cases in the world, of which nearly half are found in China. Similarly, 55% of all cancer-related fatalities occur in Asia. Researchers predicted that 8.2 million people will be diagnosed with cancer in 2018, with 5.2 million succumbing to the disease. Despite substantial research and innovations in therapeutic techniques, cancer is often detected at a late stage. It is possible to reduce the death rate at a late stage of cancer by detecting the disease at an early stage [10]. Consequently, it is a dire need to find a cancer treatment or drug candidate that is both safe and effective.

Hence, as a factor that promotes DNA replication to generate a trimeric structure, MCM7 works in conjunction with the other two members of the minichromosomal maintenance (MCM) protein family [11], a hexameric protein complex (MCM2-7). The pre-replication complex (pre-RC) that forms at the start of DNA replication is incomplete without MCM7. This led to the formation of replication forks and the utilization of numerous DNA unwinding enzymes as the pre-RC regulated helicase activity [12]. Consequently, any disruption of MCM activity results in genetic disarray and a range of carcinomas [13]. MCM7 has recently been discovered to modulate the binding activity of MCM proteins, which are strongly associated with carcinogenesis and promote cancer development [11]. MCM7 mRNA expression is a good biomarker in cervical cancer and a diagnostic biomarker in colorectal, lung, and ovarian cancer [11]. Due to the critical function of MCM7 overexpression in cancer formation, the research sought to find viable therapeutic candidates to treat human cancers. Simavastatin and Atorvastatin are reported as potential MCM7 inhibitors by suppressing RB-deficient tumor growth than the control group demonstrated by Li et al. [14].

Although, medicinal plants have a large number of useful medicinal bioactive chemicals that are beneficial against a variety of cancers [15]. These chemicals act through a variety of mechanisms and display their anticancer activity by blocking several proteins essential in cell growth and division [16]. Bioactive substances, such as small molecules, are chemical compounds or materials formed by living beings or medicinal plants that may be utilized to discover novel therapies [17]. Previously, anticancer medicines such as Taxol were derived from plant sources such as *Taxus brevifolia* and *Cinchona* spp [18]. Natural extracts are often used in anticancer medications. Herbal extracts such as ginsenoside for breast cancer [19] and ovarian cancer [20] and others have shown anti-cancer properties [21, 22]. The FDA and the European Medical Agency have authorized a quarter of plant-based medications, demonstrating their significance in the biomedical field [23]. Different medicinal plants are thought to be powerful sources of anticancer chemicals these days [24]. The traditional method of generating new pharmaceuticals is time-consuming, costly, and needs a lot of work [25]. On the contrary, drug computational design is simpler, takes less time, and needs less work [26]. The in silico high-throughput screening approach aids in the rapid generation of lead compounds at a lesser cost [27]. Furthermore, computer-aided drug design (CADD) has been used to find a varied range of prospective drug candidates utilizing a virtual screening method that combines docking, absorption, distribution, metabolism, and excretion (ADME), toxicity, and molecular dynamics (MD) simulation [28]. Trichostatin [29] A (TSA) has recently been found as a potential treatment candidate against human cancers by researchers.

The article "High-Throughput Screening and Molecular Dynamics Simulation of Natural Products for the Identification of Anticancer Agents against MCM7 Protein" was retracted in 2023. Reasons: signs of a paper mill; suspected computer-generated content; unreliable results or conclusions; concerns about the data.

As a result, the study's goal was to use computational methods to find new medication candidates that target the protein. The investigation begins by looking at the interactions between proteins and medicines. Then, utilizing virtual screening, molecular docking, ADMET, and dynamics simulation techniques, promising therapeutic candidates for proteins were found.

## 2. Methodology

### 2.1. Retrieval and Preparation of Protein

The most essential requirement for molecular docking is the presence of a 3D structure of the protein. The 3D X-ray crystalline structure of MCM7 (PDB ID: 6XTX), (UniProt ID: P33993) was derived from the Protein database with a predicted molecular weight of 81.3 kDa, a length of 719 amino acids (AA), and a resolution of 3.29 Å (Figure 1) [30]. The target MCM7 protein was co-crystallized with the MCM protein family, therefore the UCSF Chimera [31] was used to separate water, metal ions, cofactors, other compounds, and other proteins from MCM7. The UCSF Chimera was used to separate water, metal ions, cofactors, other molecules, and other proteins from MCM7, which was co-crystallized with the MCM family. AutoDock v4.2 [32] was used for further protein preparation [33]. The addition of Kollman charges, all hydrogen addition, and the fusion of non-polar hydrogen atoms are involved in the formation of the receptor [33].

The article "High-Throughput Screening and Molecular Dynamics Simulation of Natural Products for the Identification of Anticancer Agents against MCM7 Protein" was retracted in 2023. Reasons: signs of a paper mill; suspected computer-generated content; unreliable results or conclusions; concerns about the data.

### 2.2. Natural Product Compound Retrieval and Preparation

Natural product compounds were retrieved from the Natural Product Atlas library comprised of ∼29,000 compounds with referenced data for structure, total synthesis, isolation detail, organism source, and compound names [34]. It is the first comprehensive database of natural products (mainly derived from microorganisms) that can be accessed by the general public, enabling the development of new methodologies and a speedier structural characterization of vast natural product libraries. SDF files for approximately 29,000 compounds have been stored in a Bash repository on a Linux computer. The Open Babel program was used to transform the acquired 2D compound format into a 3D PDB file [35]. The FROG2 tool [36] was used to minimize the energy of the ligand library through the steepest descent algorithm using the MMFF94 force field for 1,500 steps as reported previously [37].

In addition, Gasteiger charges were added to compounds, torsion was introduced by rotating all rotatable bonds using AutoDock, and the optimized compound library was stored in PDBQT format for additional high-throughput screening.

### 2.3. Virtual Screening and Molecular Docking Studies

To investigate the inhibitory effects and binding patterns of natural product molecules, virtual screening was performed against MCM7. The docking analysis was carried out using a library of produced receptor proteins and ligands. The Lamarckian Genetic Algorithm of ADT (AutoDock) was used in this work to investigate the active binding space with varying effectiveness. The presence of a co-crystallized AGS ligand identified the binding pocket in MCM7. For docking purposes, a grid box was constructed around the receptor region where AGS had been bound [38]. The grid center settings are set to 44 points on the *x*-, *y*-, and *z*-axes, with grid center parameters set at 212.478, 230.105, and 163.638, respectively. The PDBQT library was split into the relevant file using the vina split program. Utilizing AutoDock vina v1.1.2, a maximum of 27,000 generations and 2,500,000 evaluations were possible using 250 times Lamarckian GA parameters [39].

### 2.4. ADME Profiling and Toxicity Analysis

The physiochemical attributes for the library of the natural product were studied to determine the main factors that might influence the biological activities of the lead molecules. Prediction of molecular weight, skin, cell, intestinal permeability, drug bioavailability, biopharmaceutical properties, and drug likeness are all included in the physicochemical analysis (i.e., solubility, pKa value, etc.). Furthermore, the SwissADME tool [40] was also used to assess the drug's absorption, distribution, metabolism, and excretion (ADME) capabilities, as well as several other parameters related to its pharmacological action. Furthermore, toxicity is a major problem in drug formulation. Additionally, the carcinogen pattern, Ames toxicity, and acute toxicity of rats/mouse compounds were also estimated using the SwissADME tool.

The article "High-Throughput Screening and Molecular Dynamics Simulation of Natural Products for the Identification of Anticancer Agents against MCM7 Protein" was retracted in 2023. Reasons: signs of a paper mill; suspected computer-generated content; unreliable results or conclusions; concerns about the data.

### 2.5. Molecular Dynamics Simulations

The GROMACS server v2020 [41] and published methodologies [42] MD simulations were utilized to evaluate the selected compounds' stability, binding affinity, and flexibility after docking and ADMET evaluation. The ATB v3.0 server was used to produce the ligand topology parameters. By adding solvent molecules from the SPC water model, the complex was put in a dodecahedron box with periodic boundary conditions, with the complex being positioned at a distance of 1.0 from the box border. Counter ions were introduced into a solvated solution to neutralize whole systems. When working with a maximum force of 1000 kJ mol^–1^, the neutralized system was reduced by applying the steepest descent approach. The NVT and NPT equilibration of the minimized systems was carried out for 100 ps before the production dynamics to raise the system temperature by 300 K and maintain a constant pressure of 1 bar in the system throughout the production dynamics duration. All of the bonds were restricted using the Linear Constraint Solver (LINCS) technique, and long-range electrostatics were estimated using the Particle Mesh Ewald (PME) method with a cutoff value of 1.0 nm. A 50 ns production run was completed, with coordinates and energy being collected every 10 ps in the output trajectory file, following the procedure. Additionally, the Root Mean Square Fluctuation (RMSF), Root Mean Square Deviation (RMSD), hydrogen interactions, and radius of gyration (Rg) of the system were displayed to determine its overall stability.

## 3. Results

### 3.1. Virtual Screening and Molecular Docking Studies

At the atomic level, molecular docking may anticipate a ligand's main protein-binding mode(s). Docking provides a way for virtual screening, and the result was ranked on the basis of binding scores. In molecular docking, the most efficient ligand docks minimally with its target protein and receptor protein. The binding energy of the co-crystallized AGS inhibitor was predicted to be −9.30 kcal/mol based on redocking validation which allowed the docking parameters to be employed in virtual screening with the RMSD for AGS redocking computed as 2.35 Å (Figure 2).

The article "High-Throughput Screening and Molecular Dynamics Simulation of Natural Products for the Identification of Anticancer Agents against MCM7 Protein" was retracted in 2023. Reasons: signs of a paper mill; suspected computer-generated content; unreliable results or conclusions; concerns about the data.

The structure of ~29,000 was evaluated for virtual screening utilizing Autodock Vina. Considering −9.30 kcal/mol as a cutoff value i.e., of the reference compound, virtual screening with a high throughput of utilized compounds yielded findings with acceptable high binding scores of the compounds ranging between −1 to −16.4 kcal/mol kcal/mol (Figure 3). Most compounds (*n* = 2953) were observed to have binding affinities between −7.4 to −7.9 kcal/mol (purple color). However, 1419 compounds had binding affinities <−10 kcal/mol. These compounds suggest that blocking MCM7 might be useful as a lead in the future. The top 603 compounds with binding energies <−11 kcal/mol were for further study lower than that of the reference compound, respectively.

### 3.2. ADMET-TOX and Pkscm Profiling

The substances' pharmacokinetic characteristics and toxicity profile are essential to confirm their effectiveness as well as their therapeutic and harmful effects. Pharmacokinetic (PK) features to evaluate and predict biological activities like a compound's harmful or therapeutic effect on an organism. PK properties determine whether a medication has been properly absorbed, distributed, metabolized, and removed. Based on the Blood-Brain Barrier (BBB) crossing potential, toxicological assessments, ADME profiles, and drug-likeness, the SwissADME and Pkscm online tools were used to calculate the pharmacokinetic characteristics of nominated compounds. The Lipinski rule of 5 and the CMC-like rule were used to determine the drug-likeness metric. The BBB permeability defines the ability of the compound to penetrate the CNS. The value of CNS > −2 was measured to infiltrate the Central Nervous System (CNS). Among these 603 compounds, only four compounds were selected based on their ADMET profiling i.e., NPA000018 (Lolicine A), NPA000111 (Armochaetoglobin N), NPA000305 (Quartromicin D2), and NPA014826 (Pyralomicin 2b) (Table 1).

The CNS permeability of these shortlisted compounds was −0.6, −0.5, −1.6, and 0.2, indicating that they are CNS non-accessible. In the AMES (assay to evaluate reverse mutation in *Salmonella*) and carcinogenic profile evaluation, safety and non-carcinogenicity of all four substances were expected. The Lipinski rule of five was applied to the compounds that were shortlisted (Table 2). The Lipinski rule of five was used to determine if the four lead-like compounds were in an acceptable range, as well as their pharmacokinetic and toxicological characteristics. However, NPA000111 was shown to be hepatotoxic, while NPA01478 may cause cutaneous hypersensitivity (Table 3).

The article "High-Throughput Screening and Molecular Dynamics Simulation of Natural Products for the Identification of Anticancer Agents against MCM7 Protein" was retracted in 2023. Reasons: signs of a paper mill; suspected computer-generated content; unreliable results or conclusions; concerns about the data.

### 3.3. Molecular Docking and Interaction Analysis of the Shortlisted Compounds

Compounds NPA000018, NPA000111, NPA000305, and NPA014826 have an ADMET-Tox profile that was eligible for consideration as a safe drug candidate for in-vivo research. These compounds' binding energies were calculated to be −11.9, −11.2, −11.8, and −14.2 kcal/mol, respectively. NPA014826 > NPA000018 > NPA000305 > NPA000111 was predicted as the docked compound order based on their docking score. NPA000018 was shown to mediate only one hydrogen bond inside the binding pocket of MCM7 protein, with O74 acting as a hydrogen acceptor from Lys305 with a bond length of 2.59 Å. O1 and ARG567 are linked by a hydrogen bond via NPA000111. ASP363 detected two ionic interactions, one with O2 and the other with O3 (bond lengths ranging from 1.96 nm to 3.92 nm). Arg396, Tyr403, Gln389, and Arg545 were the primary hydrophobic contacts in NPA000305 interactions via MCM7. It was revealed that NP014826 mediates one hydrogen bond as an acceptor from Arg71 through its side chain O4 atom. The 5-ring, on the other hand, had a single pi-cation interaction with Arg71, respectively (Figure 4).

The docking analysis showed that the selected four compounds had higher binding energies than the reference owing to the presence of more aromatic rings (AGS). As shown in Table 4, the interactions were mostly generated by Arg (396, 545, and 567), indicating the binding affinity of these compounds for MCM7.

### 3.4. Molecular Dynamics Simulations

The docked complex of MCM7 and the compounds (NPA000018, NPA000111, NPA000305, and NPA014826) that were identified by docking studies were further evaluated for their stability study by using MD simulation for up to 50 ns. The results of the simulation are discussed in detail concerning the radius of gyration and hydrogen bond, RMSF, and RMSD analysis.

As the RMSD values for each lead compound were within 0.3–0.45 nm, this indicates that the lead compounds found were all tightly bound inside the MCM7 active cavity. The relative motion of the protein-compound complex system remained within the RMSD range between 0.2.5 and 0.5 nm, as indicated by the RMSD graph (Figure 5(a)). The MCM7 in combination with compound NPA000018 (black) demonstrated stability after 25 ns of simulation with mild variations. At 15 ns simulation, a modest increase in the complex with NPA000111 (red) was detected causing the stability of complex after 30 ns. NPA000305 (blue), on the contrary, was optimally stable after 30 ns, resulting in the overall stability of 0.4 nm throughout this range. The NPA014874 complex (green) resulted in the steady RMSD after 15 ns with mild - to - moderate variation during the 50 ns simulations around 0.35–0.5 nm. These backbone alterations reported in MCM7 and ligand complexes imply the conformational changes as indicated by the RMSD.

The article "High-Throughput Screening and Molecular Dynamics Simulation of Natural Products for the Identification of Anticancer Agents against MCM7 Protein" was retracted in 2023. Reasons: signs of a paper mill; suspected computer-generated content; unreliable results or conclusions; concerns about the data.

The RMSF trajectories are critical to understanding the stability of the complex. Plot variations reveal how dynamics and fragile these connections are. Complex regions that are well-structured and less distorted are indicated by lower values or less variation. However, as shown in Figure 5(b), the MCM7 complex containing compounds had the same pattern of interactions throughout the system. During the entire (50 ns) simulation period, the molecules complexed with MCM7 demonstrated protein stability with mild high peaks as the consistent pattern.

In addition, the radius of gyration was investigated to determine MCM7's compactness in the presence of compounds. The simulated Rg of these four compounds is given in Figure 5(c), ranging from 2.1 to 2.2 nm. The Rg value demonstrated the protein's stability in the complex, suggesting that these four molecules are bound together without any structural changes.

Hydrogen bonding determines the strength of the interaction between ligands and proteins. Throughout the simulation, a continuous range of hydrogen bonds ~4–6 was detected in these compounds, whereas compound **NPA000018** (black) mediates 1 hydrogen bond. The NPA000111 (red) was observed to mediate ~8 bonds indicating the most stable interaction with MCM7 protein. The NPA000305 was observed to have interaction within the binding pocket of MCM7 via ~4 hydrogen bonds whereas, NPA014826 (green) formed 2-3 hydrogen bonds defining the possible significant *in silico* inhibitory activity (Figure 5(d)). During simulation, MCM7 protein was shown to be stable after 50 ns simulation of four of these compounds. Therefore, making them better options for blocking the MCM7 as a possible inhibitor.

## 4. Discussion

Cancer is one of the most lethal and preventable diseases, contributing significantly to the global number of deaths. Abnormal and unregulated cell division is the process that happens within the human body and spreads to other regions, causing tissue destruction, including the lungs, kidneys, intestines, uterus, brain, and blood, which might be affected [44]. While cancer cells multiply uncontrolled in comparison to the majority of non-cancerous cells, chemotherapy for cancer has traditionally targeted DNA replication [45]. DNA replication licensing factor and hexamer MCM (MCM2–7) complex component MCM7 (Minichromosome Maintenance Complex Component 7) control the DNA replication process. Cancer development is aided by the MCM7 protein, which is linked to tumor cell proliferation. A therapy approach for several human cancers is possible since the protein is extensively expressed during cancer development [46].

The article "High-Throughput Screening and Molecular Dynamics Simulation of Natural Products for the Identification of Anticancer Agents against MCM7 Protein" was retracted in 2023. Reasons: signs of a paper mill; suspected computer-generated content; unreliable results or conclusions; concerns about the data.

Medicinal plants have changed from fringe to mainstream usage in recent decades, and a growing number of individuals are seeking relief from herbal extracts [47]. Anti-cancer supplements have long been found in plants. Anticancer medications on the market include significant amounts of natural extracts. The anti-cancer properties of several herbal extracts [19, 20, 48], and others, have been studied extensively. These discoveries have prompted us to focus on herbal extracts in the future. For the present work, we have considered Traditional Chinese Medicine (TCM) compounds as a natural source for cancer chemotherapy. Advances in immunotherapy have transformed the treatment of several cancers. TCM which has a long history of clinical adjuvant cancer treatment, is becoming a key medical resource for developing novel cancer medicines, including immunotherapy. This study employed a quantitative and system pharmacology-based method to identify TCM-derived natural chemicals for cancer immunotherapy.

There are several advanced characteristics and procedures covered by Computer-Aided Drug Design (CADD), which is one of the most promising approaches for finding novel compounds that target specific proteins [49]. Using CADD, virtual screening may include molecular docking, ADMET, and MD simulations, reducing the time and money spent on the whole drug development process [50].

Therefore, the current study used many pharmacoinformatic-based approaches to identify potential natural product drug candidates against MCM7 protein (Figure 1) as a therapeutic option for human cancers. The research used a compressive drug design strategy to evaluate a 29,000 natural phytochemical compound library derived from microbial sources (Supplementary File 1) for their ability to combat the MCM7-related human cancers with MCM7 protein. The NPASS database is a curated natural product library that contains sufficient amounts of both active and inactive natural products. It has been widely used as novel drug candidates against SARS-CoV-2 [51, 52]. From these compounds with the greatest binding affinity as determined by the molecular docking score, the top four were selected i.e., NPA000018 (Lolicine A) (−11.9 kcal/mol), NPA000111 (Armochaetoglobin N) (−11.2 kcal/mol), NPA000305 (Quartromicin D2) (−11.8 kcal/mol), and NPA014826 (Pyralomicin 2b) (−14.2 kcal/mol) (Table 1). The ADME methods were used to study the metabolite kinetics of these molecule candidates in the body. The ADME mostly affects the pharmacokinetic parameters of the medication (Table 2). Because a prospective drug candidate has to pass a typical clinical trial, the PK parameters should be improved before the drug discovery process (Table 3). Significantly, Armochaetoglobins K-R and Quartromicin D2 are actively studied as antivirals (primarily HIV) against viral infections such as influenza virus type A, human immunodeficiency virus, and herpes simplex virus type 1 [53, 54]. Additionally, Pyralomicin is reported for its antibacterial activities [55]. Therefore, these may possess high viability as an anticancer for human cancers related to MCM7.

The article "High-Throughput Screening and Molecular Dynamics Simulation of Natural Products for the Identification of Anticancer Agents against MCM7 Protein" was retracted in 2023. Reasons: signs of a paper mill; suspected computer-generated content; unreliable results or conclusions; concerns about the data.

Moreover, it was observed that these compounds mediate interactions via ARG567, Arg71, and Lys305, while hydrophobic interactions were mainly formed through Arg396, Tyr403, Gln389, and Arg545. The docking analysis found that the four selected compounds had higher binding energies owing to more aromatic rings than the reference (AGS). Notably, Arg (396, 545, and 567) generated most of the interactions with MCM7 (Table 4). It was predicted that these four compounds were highly acceptable as drug candidates against MCM7. Importantly, a molecular simulation of these four compounds was run throughout 50 ns to examine their stability as well as the mechanism by which they inhibit MCM7. After 25 ns in the range of 3–4.5 nm, the simulation analysis shows that these four compounds with the MCM7 complex form stable complexes, which might potentially be employed in future experiments to combat human cancers linked to the MCM7 protein (Figure 5). To the best of our knowledge, this is the first complete computational investigation of possible medications from microbial natural products as candidates against human cancer that target the MCM7 protein. Although these selected compounds were potentially stable and capable of inhibiting the MCM7 protein effectively. However, testing using different lab-based trial approaches may help determine the function of the molecule, which will provide alternatives to human cancer immunotherapy.

## 5. Conclusion

MCM7, a component of the DNA replication licensing complex, is overexpressed in a variety of human malignancies. Approaches like in silico screening may give fast and accurate information on new medicinal compounds for early drug development research. Therefore, the present in silico pharmacoinformatic work reports on the pharmacological effects of a 29,000 natural product library from microbial sources against MCM7-related cancer. The four compounds that have a stronger binding affinity than AGS (reference compound): NPA000018 (−11.9 kcal/mol), NPA000111 (−11.2 kcal/mol), and NPA000305 (−11.8 kcal/mol) were shortlisted as a potent novel MCM7 inhibitor. To examine the potential of the identified compounds as therapeutic candidates against MCM7-related cancer, virtual screening, molecular docking, ADME, and toxicity investigations were conducted. MD simulations validated the biological effects of these complexes and their stability. It is expected that subsequent investigations *in vitro* and *in vivo* will revalidate these natural chemicals (primarily NPA000111 and NPA014826) as promising anticancer medicines, which need further validation in combating human malignancies.

The article "High-Throughput Screening and Molecular Dynamics Simulation of Natural Products for the Identification of Anticancer Agents against MCM7 Protein" was retracted in 2023. Reasons: signs of a paper mill; suspected computer-generated content; unreliable results or conclusions; concerns about the data.

## Figures and Tables

**Figure 1:** 3D structure of MCM7 (6XTX) integrated with AGS (red), Zn (purple), and Mn (green).

**Figure 2:** Re-docking study of MCM7 with: (a) AGS; (b) superimpose structures of AGS (magenta) and redocked (slate); (c) redocked AGS highlighted (coral arrow) in complex with MCM7.

**Figure 3:** (a) Virtual screening of 29,000 compounds, classifying compounds as mostly docked compounds (Purple), and highly docked compounds (<−10 kcal/mol); (b) identified leads like compounds (*n* = 1419); (c) and proposed leads compounds (*n* = 603) in the current study.

**Figure 4:** Docking studies of: (a) NPA000018 (Lolicine A); (b) NPA000111 (Armochaetoglobin N); (c) NPA000305 (Quartromicin D2); and (d) NPA014826 (Pyralomicin 2b) generated through the Molecular Operating Environment (MOE) tool version (MOE_2016.0802) [43].

**Figure 5:** Molecular dynamics simulation study highlighting: (a) Root Mean Square Deviation (RMSD) of the protein backbone; (b) Root Mean Square Fluctuation of proteins after simulations; (c) radius of gyration of proteins (Rg), and; (d) hydrogen bonds identified in the shortlisted compounds i.e., NPA000018 (black), NPA000111 (red), NPA000305 (blue), and NPA014826 (green).

**Table 1:** The complete detail of the shortlisted compounds.

Compound IDs	Compounds names	Origin organism	Origin genus	Origin species	Structure
NPA000018	Lolicine A	Fungi	*Neotyphodium*	*Perenne*	
NPA000111	Armochaetoglobin N	Fungi	*Chaetomium*	*Globosum* TW-1	
NPA000305	Quartromicin D2	Bacterium	*Amycolatopsis*	*Orientia* Q427-8	
NPA014826	Pyralomicin 2b	Bacterium	*Microtetraspora*	*Spiralis* MI178-39	

**Table 2:** ADME property analysis of the shortlisted compounds.

Name	Water solubility	CaCo2 permeability	HIA	Skin permeability	BBB permeability	Lipinski violation
NPA000018	−4.628	1.627	100	−2.784	No (−0.6)	Yes
NPA000111	−4.317	1.458	100	−2.785	No (−0.5)	Yes
NPA000305	−2.951	0.811	29.78	−2.735	No (−1.6)	Yes
NPA014826	−3.162	0.846	64.481	−2.757	No (−1.352)	Yes

The article "High-Throughput Screening and Molecular Dynamics Simulation of Natural Products for the Identification of Anticancer Agents against MCM7 Protein" was retracted in 2023. Reasons: signs of a paper mill; suspected computer-generated content; unreliable results or conclusions; concerns about the data.

**Table 3:** Toxicity analysis of the shortlisted four compounds.

Name	Max. tolerated dose (human)	Minnow toxicity	*T*. *Pyriformis* toxicity	Oral rat acute toxicity (LD50)	Ames test	Hepatotoxic	Skin sensitization
NPA000018	−0.265	−2.36	0.285	2.919	No	No	No
NPA000111	−0.588	0.461	0.311	2.625	No	Yes	No
NPA000305	−1.67	9.58	0.28	2.58	No	No	No
NPA014826	−0.147	2.66	0.293	2.393	No	Yes	No

**Table 4:** The interaction detail of the shortlisted compounds.

S. No.	Compounds	Name	Ligand	Receptor	Interaction	Distance	E (kcal/Mol)	S-score
1	NPA000018	Lolicine A	O 74	NZ LYS 305	H-acceptor	2.59	−2.8	−11.9
2	NPA000111	Armochaetoglobin N	O 1	NH2 ARG 567	H-acceptor	3.10	−2.2	−11.2
			O 2	OD2 ASP 363	Ionic	1.96	−16.9	
			O 3	OD2 ASP 363	Ionic	3.92	−0.7	
3	NPA000305	Quartromicin D2	Hydrophobic interactions					−11.8
4	NPA014826	Pyralomicin 2b	O 4	NE ARG71	H-acceptor	2.96	−0.8	−14.2
			5-ring	NH2 ARG71	Pi-cation	4.64	−1.0	

## Data Availability

All the data generated/analysed in the current study are available in the manuscript and supplementary files.

## Supplementary Materials

Supplementary Materials Supplementary Data File 1: Natural phytochemical compound library derived from microbial sources.
